The article "Rutin alleviates psoriasis‐related inflammation in keratinocytes by regulating the JAK2/STAT3 signaling" was published in 2024. Journal: Skin Res Technol.

# Rutin alleviates psoriasis‐related inflammation in keratinocytes by regulating the JAK2/STAT3 signaling

**DOI:** 10.1111/srt.70011

**Published:** 2024-08-21

**Authors:** Panhong Wu, Yonghui Liu, Hanxue Zhai, Xiaohan Wu, Aimin Liu

**Affiliations:** ^1^ Medical Beauty Department Henan Provincial Hospital of Traditional Chinese Medicine Zhengzhou China; ^2^ Surgery of Chinese Medicine The Second Clinical Medical College of Henan University of Traditional Chinese Medicine Zhengzhou China

**Keywords:** inflammation, keratinocytes, psoriasis, Rutin, STAT3

## Abstract

**Background:**

Psoriasis is a chronic inflammatory skin disease that can cause systemic inflammation in various organs. Rutin has been suggested to fight psoriasis, but the signaling pathways by which it works need to be explored.

**Materials and methods:**

HaCaT cells co‐stimulated with interleukin (IL)‐17, IL‐22, tumor necrosis factor‐alpha (TNF‐α), IL‐1α, and oncostatin M (M5) were used as an in vitro cell model of psoriasis. The proliferation and viability of HaCaT cells were determined by 5‐ethynyl‐2′‐deoxyuridine and cell counting assays. Relative mRNA levels of IL‐6, TNF‐α, chemokines (CXCL1 and CXCL2), and anti‐microbial peptides (S100A7 and S100A8) were detected by reverse transcriptase‐quantitative PCR. Release of IL‐6 and TNF‐α from HaCaT cells was measured by enzyme‐linked immunosorbent assay. Keratin1, Keratin5, p‐JAK2, and p‐STAT3 protein levels were estimated with western blotting. Molecular docking predicted binding sites for Rutin and STAT3.

**Results:**

Rutin treatment undercut M5‐urged viability increase and proliferation boost in HaCaT cells. Moreover, M5 stimulation mediated upregulation of IL‐6, TNF‐α, CXCL1, CXCL2, S100A7, and S100A8 was partially reversed after Rutin treatment. In addition, M5 stimulation induced downregulation of Keratin1 and Keratin5 proteins as well as upregulation of p‐JAK2 and p‐STAT3 proteins were attenuated in response to Rutin treatment, manifesting that Rutin treatment inhibited M5‐promoted aberrant differentiation and impaired M5‐mediated activation of the JAK2/STAT3 signaling in HaCaT cells. Molecular docking discovered that residues GLN326 and ASP334 in STAT3 might bind to Rutin.

**Conclusion:**

Rutin treatment blocked the JAK2/STAT3 signaling, thus attenuating psoriasis‐related inflammation and anomalous differentiation in keratinocytes.

## 1 INTRODUCTION

Psoriasis is a chronic immune‐mediated inflammatory disease that affects approximately 60 million people worldwide.^1^, ^2^ Psoriasis presents as red and scaly plaques which are frequently observed on the lower back, elbows, knees, and scalp.^3^ Skin involvement is the main feature of the disease, but it may also cause systemic inflammation in various organs.^4^ Dendritic cells are the most important innate immune activators in psoriasis pathogenesis.^5^ Activated plasmacytoid dendritic cells by genetic and/or environmental factors produce large amounts of pro‐inflammatory cytokines [(such as interleukin (IL)‐17, IL‐22, IL‐23, IL‐1β, interferon (IFN)‐γ, and tumor necrosis factor (TNF)‐α], which can then trigger the onset of psoriasis.^6^ These cytokines compel hyperproliferation and aberrant differentiation of keratinocytes, causing the cells to produce a variety of cytokines, chemokines, and anti‐microbial peptides, which promotes a sustained pro‐inflammatory response.^7^ Existing therapies for psoriasis provide temporary symptomatic relief rather than a cure, focusing on the use of monoclonal antibodies (such as anti‐IL‐17 antibody) and immunosuppressive drugs (such as cyclosporine).^8^ Therefore, the development of new strategies for curing the disease or relieving its symptoms in the long‐term is urgently needed.

The article "Rutin alleviates psoriasis‐related inflammation in keratinocytes by regulating the JAK2/STAT3 signaling" was published in 2024. Journal: Skin Res Technol.

Recently, bioflavonoids have been applied in the healthcare system, thanks to their wide range of biological activities, low cost, and high safety profile.^9^ Rutin (also called quercetin‐3‐rutinoside) is a polyphenolic bioflavonoid whose natural sources are fruits, herbs, and plants.^10^ Currently, several pharmacological properties of Rutin have been demonstrated, such as antihypertensive, hypolipidemic, antiallergic, cytoprotective, anti‐inflammatory, and anti‐viral.^11^ Peres et al. uncovered that Rutin has a distinct anti‐oxidant potential in dermocosmetic preparations.^12^ Specifically, Rutin‐mediated anti‐inflammatory activity has been reported in several chronic inflammatory diseases, including rheumatoid arthritis^13^ and multiple sclerosis.^14^ As a potent anti‐inflammatory agent, Rutin has a potentially protective role in psoriasis,^15^ but the signaling pathways by which it works need to be validated and explored.

In the current research, we used HaCaT cells stimulated with a panel of pro‐inflammatory cytokines as an in vitro cell model of psoriasis to characterize the role of Rutin and its associated pathways in psoriasis, providing evidence in support of Rutin as a potential therapeutic agent for psoriasis.

## 2 MATERIALS AND METHODS

### 2.1 Cell culture

Human keratinocytes HaCaT (Cat#C6282, Beyotime, Shanghai, China) were cultured in a complete medium (Cat#C6282C, Beyotime) at 37°C with 5% CO_2_. For simulating psoriasis conditions in vitro, HaCaT cells were synchronously stimulated for 24 h with 5 pro‐inflammatory cytokines IL‐17A (Cat#LT0125, LetoZyme, Beijing, China), IL‐22 (Cat#P5228, Beyotime), TNF‐α (Cat#LT0212, LetoZyme), IL‐1α (Cat#LT0110, LetoZyme), and oncostatin M (Cat#P5358, Beyotime) (M5), with the concentration of each cytokine at 10 ng/mL.^16^ For Rutin treatment, HaCaT cells were incubated in a complete medium with different concentrations of Rutin (0, 1, 5, 10, 15, 30, 50, and 100 μM) (Cat#HY‐N0148, MCE, New Jersey, USA) for 2 h prior to stimulation with M5, with dimethyl sulfoxide as a solvent.

The article "Rutin alleviates psoriasis‐related inflammation in keratinocytes by regulating the JAK2/STAT3 signaling" was published in 2024. Journal: Skin Res Technol.

### 2.2 Cell counting kit‐8 (CCK‐8) assays

HaCaT cells (5×10^3^ cells/well) were cultured for 24 h in different groups. Ten microliters of the CCK‐8 solution (Cat#C0038, Beyotime) were added to each well and incubation was continued for 2 h. Spectro colorimetric analysis was executed with a microplate reader (450 nm, Tecan, Mannedorf, Switzerland). Calculation of cell viability was accomplished using the following equation: cell viability (%) = (OD_experimental_‐OD_background_/OD_control_‐OD_background_) × 100 %.

### 2.3 5‐ethynyl‐2′‐deoxyuridine (EdU) labeling assays

HaCaT cells (2.5×10^5^ cells/well) were treated in different groups for 24 h, followed by incubating with EdU (Cat#CX002, 10 µM, Cellorlab, Shanghai, China) for 3 h. After digestion with 0.25% trypsin (Cat#9002‐07‐7, Targetmol, Shanghai, China), HaCaT cells were fixed with 4% paraformaldehyde (Cat#P0099, Beyotime), permeabilized with 0.3% Triton X‐100 (Cat#9002‐93‐1, Targetmol), and stained with a click reaction solution (Cat#CX002, Cellorlab) for 30 min. Staining of nuclei was carried out with 100 µL of 4′,6‐diamidino‐2‐phenylindole (Dapi) (Cat#C1002, Beyotime) for 30 min. Proportion of EdU‐incorporated cells was estimated using a fluorescence microscope (Olympus, Tokyo, Japan).

### 2.4 Western blotting

HaCaT cells with different treatments were subjected to protein extraction via the radioimmunoprecipitation assay method (Cat#PC101, Cellorlab). Equal amounts of proteins were subjected to sodium dodecyl sulfate‐polyacrylamide gel electrophoresis and then transferred to a polyvinylidene difluoride membrane. Subsequently, the membrane underwent blocking, followed by detection with specific primary antibodies, including Keratin5 (Cat#GTX11321, 1:1000, GeneTex, Irvine, CA, USA), Keratin1 (Cat#M01639‐1, 1:5000, BosterBio, Wuhan, China), p‐Janus kinase 2 (JAK2) (Cat#GTX132784, 1:1000, GeneTex), p‐signal transducer and activator of transcription 3 (STAT3) (Cat#bs‐55208R, 1:1000, Bioss, Beijing, China), and β‐actin (Cat#ab8226, 1:10 000, Abcam, Cambridge, Massachusetts, USA). Following incubation with an appropriate secondary antibody, protein bands were visualized using a high‐signal ECL western blotting substrate (Cat#E411‐04, Vazyme, Nanjing, China), and gray‐scale values of all bands were obtained using ImageJ (NIH, Bethesda, Maryland, USA), and relative protein expression levels were determined using β‐actin as a standard.

The article "Rutin alleviates psoriasis‐related inflammation in keratinocytes by regulating the JAK2/STAT3 signaling" was published in 2024. Journal: Skin Res Technol.

### 2.5 Reverse transcriptase‐quantitative PCR (RT‐qPCR)

Total RNA of HaCaT cells cultured in different groups was extracted using the VeZol‐pure total RNA isolation kit (Cat#RC202‐01, Vazyme) as per the manufacturer's protocol. Measurement of the concentration of extracted RNA was made with a NanoDrop 2000 Lite spectrophotometer (Thermo, Waltham, Massachusetts, USA). Total RNA (1 µg) was converted to complementary DNA by HiScript II Q RT SuperMix for qPCR (+gDNA wiper) (Cat#R223‐01, Vazyme). Quantitative PCR was performed by using AceQ qPCR SYBR green master mix (Cat#Q111‐02, Vazyme). Relative mRNA expression levels were calculated using the 2^−ΔΔCT^ method^17^ and normalized to the glyceraldehyde‐3‐phosphate dehydrogenase.

### 2.6 Enzyme‐linked immunosorbent assay (ELISA)

HaCaT cells with different treatments were cultured for 24 h. The release of IL‐6 and TNF‐α from HaCaT cells was determined using specific ELISA kits (Cat#EMT2010‐1, Assaypro, St. Charles, Missouri, USA; Cat# FEK0411, BosterBio). Measurement was conducted at 450 nm using a microplate reader (Tecan).

### 2.7 Molecular docking

A molecular docking assessment was performed to determine the binding affinity of Rutin toward STAT3. The structure of Rutin was obtained by Pubchem (https://pubchem.ncbi.nlm.nih.gov/compound/5280805). For the three‐dimensional structure of STAT3, it was obtained from the Protein Data Bank database (https://www.uniprot.org/). By utilizing the AutoDock 4.2 software, the binding sites between Rutin and STAT3 were predicted. Visualization of docking results was performed using PyMol 2.2.

### 2.8 Data analysis

All experiments were performed in triplicate with at least three biological replicates. Data were shown as mean and standard error mean. Statistical analysis was calculated by Prism 9 (GraphPad Software, USA). Tests for differences among multiple populations were conducted with analysis of variance (ANOVA) with Dunnet's post‐hoc test. A *p*‐value of less than 0.05 was considered significant.

## 3 RESULTS

### 3.1 Rutin restrained the abnormal proliferation but not the survival of M5‐treated HaCaT cells

Rutin is a natural flavonoid glycoside with anti‐inflammatory properties, whose chemical structure (molecular formula: C_27_H_30_O_16_) is shown in Figure 1A. Inflammatory responses associated with psoriasis have been shown to be mitigated by Rutin, but the role of Rutin in psoriasis still needs to be further investigated. Here, we first estimated the cytotoxicity of Rutin on normal keratinocytes. CCK‐8 assays showed that Rutin exhibited a suppressive influence on HaCaT cell viability at concentrations up to 50 µM, whereas 100 µM was close to the semi‐inhibitory concentration (Figure 1B). Based on safety considerations, we chose 10  and 30 µM for subsequent experiments. Subsequently, HaCaT cells were then co‐stimulated with M5 to mimic psoriasis in vitro. As expected, M5 stimulation elevated cell viability and facilitated cell proliferation in HaCaT cells, but Rutin treatment restrained HaCaT cell viability and proliferation under M5 stimulation (Figure 1C, D). These results manifested that Rutin could suppress the proliferation but not the survival of M5‐treated HaCaT cells.

The article "Rutin alleviates psoriasis‐related inflammation in keratinocytes by regulating the JAK2/STAT3 signaling" was published in 2024. Journal: Skin Res Technol.

**FIGURE 1:** Rutin could repress the proliferation but not the survival of HaCaT cells following M5 stimulation. (A) The chemical structure of Rutin (molecular formula: C27H30O16). (B) CCK‐8 assays evaluated the cytotoxicity of different concentrations of Rutin (0, 1, 5, 10, 15, 30, 50, and 100 µM) on HaCaT cells. ^**^ *p *< 0.01 and ^***^ *p *< 0.01 vs. 0 µM. (C and D) CCK‐8 and EdU assays determined the viability and proliferation of M5‐stimulated HaCaT cells and Rutin‐treated M5‐stimulated HaCaT cells. ^***^ *p *< 0.001 vs. control; ^##^ *p *< 0.01 and ^###^ *p *< 0.001 vs. M5. The data were compared by ANOVA.

### 3.2 Rutin contributed to the differentiation of M5‐stimulated HaCaT cells

Considering that the decreased terminal differentiation capacity of keratinocytes is a phenotypic feature of psoriatic lesions,^18^ we further characterized the effect of Rutin on the differentiation capacity of M5‐stimulated HaCaT cells by detecting the keratinocyte differentiation markers Keratin1 and Keratin5. The results showed that Keratin1 and Keratin5 protein levels were decreased in M5‐stimulated HaCaT cells compared to control cells, but these decreased protein levels were partially reversed upon Rutin treatment (Figure 2A‐C). These outcomes suggested that Rutin could ameliorate M5‐induced aberrant differentiation of HaCaT cells.

**FIGURE 2:** M5‐induced abnormal differentiation of HaCaT cells was ameliorated following Rutin treatment. (A–C) Western blotting assessed the protein levels of Keratin1 and Keratin5 in M5‐stimulated HaCaT cells and Rutin‐treated M5‐stimulated HaCaT cells. ^***^ *p *< 0.001 vs. control; ^##^ *p *< 0.01 and ^###^ *p *< 0.001 vs. M5. Differential expression testing was performed with ANOVA.

### 3.3 Rutin repressed the inflammatory response of M5‐treated HaCaT cells

Because psoriasis is a chronic inflammatory skin disease, we further analyzed the influence of Rutin on psoriasis‐associated inflammation. RT‐qPCR showed that Rutin treatment weakened M5‐mediated upregulation of IL‐6 and TNF‐α mRNA levels in HaCaT Cells (Figure 3A, B). Consistently, M5‐induced release of IL‐6 and TNF‐α was also attenuated by Rutin treatment (Figure 3C, D). As for the chemokines C‐X‐C motif chemokine ligand (CXCL) 1 and CXCL2, their mRNA levels were also upregulated after M5 stimulation, whereas Rutin treatment reversed M5 stimulation‐mediated effects on CXCL1 and CXCL2 mRNA levels (Figure 3E, F). Studies have shown that anti‐microbial peptides secreted by keratinocytes are associated with the severity of psoriatic lesions.^19^ Therefore, we explored the effect of Rutin on the anti‐microbial peptides S100A7 and S100A8. Data showed that M5 stimulation significantly enhanced S100A7 and S100A8 mRNA levels, whereas M5‐mediated upregulation of S100A7 and S100A8 mRNA levels was diminished post‐treatment with Rutin (Figure 3G, H). Collectively, these results suggested that Rutin treatment decreased the inflammatory response of M5‐treated HaCaT Cells.

The article "Rutin alleviates psoriasis‐related inflammation in keratinocytes by regulating the JAK2/STAT3 signaling" was published in 2024. Journal: Skin Res Technol.

**FIGURE 3:** Treatment with Rutin reduced M5‐induced inflammatory response in HaCaT Cells. (A and B) RT‐qPCR evaluated IL‐6 and TNF‐α mRNA levels in M5‐stimulated HaCaT cells and Rutin‐treated M5‐stimulated HaCaT cells. ^***^ *p *< 0.001 vs. control; ^#^ *p *< 0.05, ^##^ *p *< 0.01, and ^###^ *p *< 0.001 vs. M5. (C and D) ELISA measured the release of IL‐6 and TNF‐α from the above‐mentioned HaCaT cells. ^***^ *p *< 0.001 vs. control; ^#^ *p *< 0.05, ^##^ *p *< 0.01, and ^###^ *p *< 0.001 vs. M5. (E‐H) RT‐qPCR detected the mRNA levels of CXCL1, CXCL2, S100A7, and S100A8 in the above‐mentioned HaCaT cells. ^***^ *p *< 0.001 vs. control; ^#^ *p *< 0.05, ^##^ *p *< 0.01, and ^###^ *p *< 0.001 vs. M5. Statistical differences were analyzed using ANOVA.

### 3.4 Rutin suppressed the JAK2/STAT3 signaling in M5‐treated HaCaT cells

Available evidence suggests that cytokines in the JAK/STAT pathway play a crucial role in common skin diseases, including psoriasis.^20^ Here, we further uncovered whether Rutin can control the JAK2/STAT3 signaling in M5‐treated HaCaT cells. The results manifested that stimulation with M5 significantly elevated the protein levels of p‐JAK2 and p‐STAT3 in HaCaT cells, but the addition of Rutin weakened M5‐induced upregulation of p‐JAK2 and p‐STAT3 protein levels (Figure 4A‐C). Application of computer‐simulated molecular docking revealed that residues GLN326 and ASP334 in STAT3 might bind to Rutin, suggesting that Rutin may exert its effects by targeting STAT3 (Figure 4D). These data manifested that Rutin might target STAT3 to suppress the JAK2/STAT3 signaling in M5‐treated HaCaT cells.

**FIGURE 4:** Rutin repressed the JAK2/STAT3 signaling in M5‐treated HaCaT Cells. (A–C) Relative protein levels of p‐JAK2 and p‐STAT3 in M5‐stimulated HaCaT cells and Rutin‐treated M5‐stimulated HaCaT cells were estimated by western blotting. ^***^ *p *< 0.001 vs. control; ^#^ *p *< 0.05, ^##^ *p *< 0.01, and ^###^ *p *< 0.001 vs. M5; ns: not significant (*p *> 0.05). Statistical differences were estimated by ANOVA. (D) Structural demonstration of the predicted binding mode of Rutin to STAT3.

The article "Rutin alleviates psoriasis‐related inflammation in keratinocytes by regulating the JAK2/STAT3 signaling" was published in 2024. Journal: Skin Res Technol.

## 4 DISCUSSION

A well‐functioning skin barrier is essential for maintaining healthy skin, and various botanical agents have been demonstrated to possess therapeutic potential in many skin barrier disorders in recent years.^21^, ^22^, ^23^, ^24^ Psoriasis, a prevalent papulosquamous skin disease worldwide, can cause skin symptoms, psychological abnormalities, and joint pathology. Therefore, exploration of novel botanical agents to alleviate the skin barrier disruption associated with psoriasis is necessary. Evidence to date has demonstrated that the prevention of inflammation‐related damage is a definitive and attainable therapeutic goal for psoriasis.^4^ It is well established that Rutin is effective against multiple inflammatory diseases, including psoriasis.^25^, ^26^ Although Rutin attenuates inflammation associated with psoriasis,^26^ the mechanisms mediated by which Rutin exerts its effects are unclear. Here, we demonstrated that Rutin mitigated psoriasis‐associated inflammation by inactivating the JAK2/STAT3 signaling.

A mixture of M5 cytokines was able to induce keratinocytes to exhibit several features of psoriatic keratinocytes,^27^ and many studies have used M5 cytokine mixtures to establish an in vitro model of psoriatic keratinocytes.^28^, ^29^ The present study established an in vitro cell model of psoriasis by stimulating HaCaT cells with 10 ng/mL of M5 to investigate the role of Rutin and its associated signaling pathways.

Keratinocytes are not only an important component in maintaining skin structure but also a major player in the skin's immune system. Multiple inflammatory mediators in psoriasis‐affected lesions act directly or indirectly on keratinocytes, leading to hyperproliferation and activation of keratinocytes. Moreover, keratinocytes recruit T cells and neutrophils by secreting IL‐6 and TNF‐α, chemokines, and anti‐microbial peptides, thereby contributing to dermal infiltration. The neutrophil chemokines CXCL1 and CXCL2 released by keratinocytes can further exacerbate inflammation by acting on vascular endothelial cells and mast cells to reactivate the central granulocyte axis. Thus, targeting the inflammation of keratinocytes is crucial for psoriasis. Recent studies found that Rutin can alleviate psoriasis. Lang et al. uncovered that Rutin could lessen oxidative stress injury induced by H_2_O_2_ in HaCaT cells through the Nrf2 signaling.^26^ Wang et al. exposed that the inflammatory response in psoriasis was lessened by Rutin through inactivating the AGE/RAGE signaling.^30^ Here, our results exhibited that Rutin treatment relieved M5‐induced viability elevation and proliferation promotion for HaCaT cells. Moreover, M5‐induced elevation of chemokines (CXCL1 and CXCL2), pro‐inflammatory cytokines (IL‐6 and TNF‐α), and anti‐microbial peptides (S100A7 and S100A8) were partly reversed following Rutin treatment, suggesting that Rutin treatment could mitigate psoriasis‐related inflammation.

The article "Rutin alleviates psoriasis‐related inflammation in keratinocytes by regulating the JAK2/STAT3 signaling" was published in 2024. Journal: Skin Res Technol.

Keratin is the major structural protein of keratinocytes, maintaining the structural stability and integrity of keratinocytes.^31^ Abnormal expression of keratins is associated with a variety of skin diseases, and changes in keratin expression may cause incomplete differentiation of epidermal keratinocytes, leading to skin hyperplasia.^32^ Roth et al. reported that Keratin1 has an important role in the maintenance of skin integrity, and it is involved in the skin inflammatory network by mediating IL‐18.^33^ Abnormal keratin5 expression impairs the structure and function of the basal cell keratin cytoskeleton, leading to skin fragility.^34^ Here, we observed that the inhibitory effects of M5 cytokines on Keratin1 and Keratin5 were impaired upon Rutin treatment, manifesting that Rutin treatment eased the abnormal differentiation of keratinocytes in psoriasis.

The JAK/STAT signaling is affected by a variety of growth factors and cytokines, participating in many important biological processes, such as cell apoptosis, proliferation, differentiation, and immunomodulation.^35^ Studies have shown that various herbal monomers or active ingredients may be involved in psoriasis by modulating the JAK/STAT signaling.^36^ For instance, kaempferol improved psoriasis by modulating IFN‐γ‐induced the JAK/STAT signaling.^37^ Total glucosides of paeony repressed the phosphorylation of STAT1 and STAT3, thus attenuating animal psoriasis.^38^ Centella asiatica blocked the JAK/STAT3 signaling, resulting in alleviating psoriasis.^39^ STAT3 is a key player in psoriasis pathogenesis and psoriasiform inflammation.^40^ STAT3 activation in psoriatic keratinocytes is caused by phosphorylation of Tyr705 in STAT3 by stimulation of pro‐inflammatory factors.^41^ A study showed that a strong increase in STAT3 transcriptional activity resulted from JAK2‐dependent phosphorylation of Tyr705 mediated by IL‐20 and IL‐6.^42^ Here, the upregulation of p‐JAK2 and p‐STAT3 mediated by M5 stimulation in HaCaT Cells was undercut following Rutin treatment. Notably, computer‐simulated molecular docking displayed that residues GLN326 and ASP334 in the DNA‐binding domain (DBD) structural domain of STAT3 might bind to Rutin. The DBD domain of STAT3 helps to recognize and bind to its target DNA‐GAS sequence.^43^ Also, the DBD domain is a “druggable” domain in STAT3, and interfering with DBD activity can directly inhibit the interaction of STAT3 with its target double‐stranded DNA.^44^ Therefore, we inferred that Rutin may work by binding to residues GLN326 and ASP334 in STAT3 to inhibit the interaction of STAT3 with its target double‐stranded DNA. All outcomes manifested that Rutin might exert its role in M5‐stimulated HaCaT Cells through controlling the JAK2/STAT3 signaling. The limitations of this study are as follows: (1) it was not verified whether STAT3 is a target of Rutin; (2) it was not verified that Rutin is effective against psoriasis by targeting STAT3 through animal models with psoriatic lesions. The above‐mentioned limitations are the direction of our further research.

The article "Rutin alleviates psoriasis‐related inflammation in keratinocytes by regulating the JAK2/STAT3 signaling" was published in 2024. Journal: Skin Res Technol.

## 5 CONCLUSION

Rutin could lighten M5‐induced inflammation and abnormal differentiation in HaCaT cells by mediating the JAK2/STAT3 signaling, which offers evidence to bolster the potential of Rutin as a drug for managing psoriasis.

## CONFLICT OF INTEREST STATEMENT

The authors declare that they have no competing interests.

## ETHICS STATEMENT

This article does not contain any studies with human or animal subjects performed by any of the authors.

## Data Availability

The data that support the findings of this study are available from the corresponding author upon reasonable request.
